RETRACTED

# Inhibition of TNF-*α* and JNK Signaling Pathway Can Reduce Paclitaxel-Induced Apoptosis of Mouse Cardiomyocytes

**DOI:** 10.1155/2022/8460121

**Published:** 2022-08-16

**Authors:** Shuang Ren, Tianwen Huang, Danyan Ou, Luhuai Feng, Sisi Huang, Chaonan Zhou, Lianying Ge

**Affiliations:** ^1^Department of General Internal Medicine, Guangxi Medical University Cancer Hospital, Nanning, 530021 Guangxi, China; ^2^Department of Clinical Pharmacy, Guangxi Medical University Cancer Hospital, Nanning, 530021 Guangxi, China; ^3^Ultrasonic Department, Guangxi Medical University Cancer Hospital, Nanning, 530021 Guangxi, China

## Abstract

Paclitaxel (PTX) is a widely used chemotherapeutic drug for treating tumors. However, studies have shown that it can cause cardiac problems such as arrhythmia, myocarditis, chronic cardiomyopathy, and heart failure. Therefore, it is essential to study the mechanism behind the cardiotoxicity of PTX in tumor treatment. In this study, we initially injected PTX into mice to establish a myocardial cell apoptosis model to observe the degree of damage to mouse myocardium caused by PTX. Upon determining the levels of mouse myocardial creatine phosphokinase (CK), myokinase isoenzyme (CK-MB), aspartate transaminase (AST), and lactate dehydrogenase (LDH), we found that all of these levels showed apparent increases in mice treated with PTX. Further analyses of the TNF-*α* level and the expression of Jun N-terminal kinase (JNK) and Bcl-2 family-related proteins in myocardial tissue were performed. It was found that PTX increased the protein levels of TNF-*α*, Bax, p-JNK, and JNK in myocardial tissue but decreased the protein level of Bcl-2. After 1 month of PTX treatment in mice, we inhibited the expression of TNF-*α* and JNK proteins, which reduced the effect of paclitaxel on the apoptosis of mouse cardiomyocytes. The protein levels of Bax, p-JNK, and TNF-*α* in cardiomyocytes were reduced, while there was a relative increase in the Bcl-2 protein level. The findings suggested that inhibition of the NK signaling pathway and TNF-*α* can lessen the effect of PTX on mouse cardiomyocytes.

## 1. Introduction

Continuous improvements in tumor treatment efficacy have prolonged patient survival [1]. The primary tumor treatment options are chemotherapy, targeted therapy, and immunotherapy [2, 3]. However, it has been reported that chemotherapy and targeted drugs can increase the risk of heart damage [4, 5]. McGowan et al. [6] stated that cancer patients treated with many anthracyclines might become tomorrow's heart disease patients. Trastuzumab is also a molecular-targeted drug most widely reported to be associated with cardiotoxicity [7, 8]. Among antimicrotubule chemotherapy drugs, docetaxel and paclitaxel can also induce cardiotoxicity (arrhythmia, sinus bradycardia, etc.) [9, 10].

RETRACTED

Paclitaxel (PTX) is a drug extracted from yew that exerts effects against various tumors. It is one of the antitumor drugs most widely used in chemotherapy during the past 20 years, including for head and neck malignancies, lung malignancies, breast malignancies, endometrial malignancies, cervical malignancies, and colorectal cancers. It has various activities in several malignant tumors [11]. Cardiotoxicity of PTX is relatively rare, but it has been reported that the drug can cause heart problems such as myocarditis [12] and heart failure [13]. It also reduces the heart function and quality of life of patients. Therefore, studying the toxic effects and mechanisms of action of PTX on the heart and then taking adequate measures to reduce the occurrence of heart disease is very important in tumor treatment.

It has been reported that oxidative stress, ischemia/reperfusion, and other factors can induce the apoptosis of myocardial cells [14, 15], which can lead to various cardiovascular diseases. Therefore, reducing cardiomyocyte apoptosis is one of the most important targets for treating cardiovascular diseases. The c-Jun N-terminal kinase (JNK) pathway is a subclass of the MAPK (mitogen-activated protein kinase) pathway, which is involved in various biological processes such as the cell cycle, growth, apoptosis, and cell stress [16].

A series of proteins in the cell called the MAPK/ERK pathway sometimes referred to as the Ras-Raf-MEK-ERK pathway and transmits signals from a receptor on the cell's surface to the DNA inside the nucleus of the cell. In eukaryotes, which include yeast and humans, MAPK modules comprised of 3 sequentially activated protein kinases are essential to several signal transduction pathways that control activities, including cell division, proliferation, and death [17]. There are three families of MAP kinases. These are ERKs (extracellular-signal-regulated kinases), JNKs, and p38/SAPKs (stress-activated protein kinases) in mammals [18]. JNK is activated and transferred to the nucleus, stimulating the transcription factor c-Jun and its phosphorylation, promoting apoptosis, and differentiation [19]. Tumor necrosis factor-alpha (TNF-*α*) is an essential regulator of apoptosis and inflammation. It promotes apoptosis by binding to TNF receptor 1 [20]. It is necessary to investigate further the JNK signaling pathway and TNF-*α* to safeguard cardiomyocytes. Therefore, this work is aimed at examining the impact of TNF-*α* and the JNK signaling pathway on the cardiomyocytes of PTX-treated mice.

## 2. Materials and Methods

### 2.1. Laboratory Animals and Reagents

Forty healthy, clean mice weighing between 18 and 22 g were purchased from the Animal Center of Guangxi Medical University. The TNF-*α* ELISA kit was purchased from Biovision (product number K1052-100). JNK, TNF-*α*, p-JNK, Bcl-2, Bax, and *β*-actin antibodies were purchased from Yubo Biotechnology Co., Ltd. HRP goat anti-rabbit IgG was purchased from Boaosen Biotechnology. ECL color development kit was purchased from Shanghai Yisheng Biotechnology Co., Ltd. BCA kits and protein extraction kits were purchased from Image Technology Co., Ltd. Trypsin, dimethyl sulfoxide, and fetal bovine serum were all purchased from Sigma (USA). DMEM was purchased from Beijing Kairuiji Biotechnology Co., Ltd.

RETRACTED

### 2.2. Experimental Grouping and PTX Intervention

The 40 mice were divided into a blank control group, PTX 50*μ*g/50g group, PTX 100*μ*g/50g group, and PTX 150*μ*g/50g group, with 10 mice in each group. The PTX in the 50*μ*g/50g group was diluted with physiological saline to 0.5*μ*g/*μ*L; so, the actual dose used was 0.5*μ*g/*μ*L × 100*μ*L = 50*μ*g/50g body weight. The PTX in the 100*μ*g/50g group was diluted with physiological saline to 1.0*μ*g/*μ*L; so, the actual dose used was 1.0*μ*g/*μ*L × 100*μ*L = 100*μ*g/50g body weight. The PTX in the 150*μ*g/50g group was diluted to 1.5*μ*g/*μ*L with saline; so, the actual dose used was 1.5*μ*g/*μ*L × 100*μ*L = 150*μ*g/50g body weight. These interventions were performed by intraperitoneal injection every 3 days for 3 months.

### 2.3. Detection of Myocardial Enzyme Indexes and Serum TNF-*α* Changes in Mice

After 3 months of PTX intervention, 2mL of blood was taken from the eyeballs of the mice and collected in EP (Eppendorf) tubes. After the blood was allowed to stand for 2 h, it was centrifuged at 12,000rpm for 10 min, and then the supernatant was obtained. The TNF-*α* level was detected using a TNF-*α* ELISA kit. The mice were sacrificed, after which the thoracic cavity was quickly opened to take blood from the heart. If the amount of blood collected was too small because the heart stopped beating, large blood vessels were cut open for further collection. The collected blood was immediately sent to the laboratory for determination of the levels of the myocardial enzymes creatine phosphokinase (CK), myokinase isoenzyme (CK-MB), and aspartate aminotransferase (AST), and lactate dehydrogenase (LDH).

### 2.4. Detection of the Protein Levels of JNK, Bax, p-JNK, and Bcl-2 in Myocardial Tissue

Myocardial tissue was dissolved with RIPA lysis buffer, and total protein was extracted through the BCA kit (Image Technology Co., Ltd, Sigma Aldrich, USA). The protein loading volume was 60*μ*g. The protein was separated by SDS-PAGE electrophoresis, followed by transfer to a nitrocellulose membrane. The nitrocellulose membrane was sealed with 5% skim milk for 1.5h, after which p-JNK (1 : 800), JNK (1 : 800), TNF-*α* (1 : 800), Bax (1 : 800), Bcl-2 (1 : 800), and *β*-actin (1 : 1,000) primary antibodies were each added, followed by incubation for 12 h. Then, an HRP-labeled goat anti-mouse secondary antibody (1 : 5,000) was added, followed by incubation for 1.5 h. Hypersensitive ECL (Enhanced chemiluminescence) liquid was added to react with the blot in the dark for 5 min. A gel imaging system was used to obtain photographs, and ImageJ software was used to analyze each protein band's intensity level.

RETRACTED

### 2.5. Nano-PCR (Polymerase Chain Reaction) Detection

TRIzol Reagent was used to extract total cellular RNA, which was then reverse-transcribed into cDNA using a reverse-transcription kit. The PCR reaction system included 10 *μ*L of 2× SYBR Premix Taq II, 0.4 *μ*L of upstream primer, 0.4 *μ*L of reverse primer, and 2 *μ*L of cDNA template, with DEPC (diethylpyrocarbonate) water added to make up the volume to 20 *μ*L. A total of 0.5 *μ*M/20 *μ*L of gold nanoparticles were added to the above reaction system. Gold nanoparticles can gather droplets on the top of the centrifuge tube to form nanodroplets, which accelerate the rate of temperature conduction from the top cover of the PCR instrument to the temperature in the reaction system. This improves the sensitivity and detection accuracy of the PCR reaction. The PCR amplification program was as follows: 95°C preheating for 1 min, 35 cycles of 30 s denaturation at 94°C, 30 s renaturation at 60°C, 1 min extension at 72°C, and finally, maintenance at 72°C for 5 min. GAPDH was used as a reference gene, and the expression level was calculated using the formula 2^–△△Ct^.

### 2.6. Inhibition of JNK and TNF-*α*

Mice in the PTX 50 *μ*g/50 g group, PTX 100 *μ*g/50 g group, and PTX 150 *μ*g/50 g group were treated with PTX for 1 month, followed by the oral JNK inhibitor JNK-IN-8 (MedChemExpress) and the TNF-*α* inhibitor TNF-*α*-IN-1 (MedChemExpress) for 2 months.

### 2.7. TUNEL Staining to Detect Cardiomyocyte Apoptosis

Frozen myocardial tissue sections were fixed with 10% neutral formaldehyde for 10 min and rinsed with PBS. The sections were then put in an acetic acid solution: ethanol (1 : 2), reacted at –20°C for 5 min, and washed with PBS for 10 min. PBS containing 2% H_2_O_2_ was added to the slices, followed by a reaction at room temperature for 5 min, and washed with PBS. Two drops of TdT (terminal deoxynucleotidyl transferase) enzyme buffer was added and allowed to react for 3 min at 25°C. Afterward, 50 *μ*L of TdT enzyme reaction solution was added and allowed to react at 37°C with 50% humidity for 1 h. Then, the slices were placed on a staining plate with a washing buffer and a stop reaction buffer, and the mixture was left to react for 30 min at 37°C. Two drops of antidigoxin antibody were applied dropwise and left to react for 0.5 hr at 25°C with 50% humidity after the sections had been rinsed with PBS for 15 min.

RETRACTED

Subsequently, the sections were washed with PBS for 20 min, and the newly prepared 0.05% DAB (3,3′-diaminobenzidine) solution was added dropwise. The color was produced for 3 to 6 min at 25°C, washed for 8 min in distilled water, and redyed for 10 min in methyl green. The slides were put in distilled water for 30 s after being submerged for 1 s. Then, the slides were lifted, and this step was repeated 20 times. Following this, the slide glass was immersed for 30 s after submerging in 100% n-butanol and raised 20 times. The slices were then dehydrated with xylene 3 times for 2 min each. After mounting and drying the slides, the results were examined under a microscope.

### 2.8. Statistical Analysis

Comparisons between the groups were performed using SPSS 21.0 and GraphPad Prism statistical software. Data are shown as mean ± standard deviation. The *t*-test was used for comparing two groups, while variance analysis (ANOVA) was used for multigroup comparisons. Differences were found to be statistically significant if *P* < 0.05.

## 3. Results

### 3.1. Changes in Myocardial Enzyme Indexes and Serum TNF-*α* in Mice after PTX Intervention

When cardiomyocytes become necrotic for various reasons, their enzymes enter the blood, increasing the blood enzyme level [21]. This study evaluated the damage caused by different concentrations of PTX to mouse myocardium. By detecting the levels of mouse myocardial enzymes, we found that, after treatment with PTX, the myocardial enzymes CK, CK-MB, and AST and the average expression level of LDH increased markedly (*P* < 0.05, Figures 1(a)–1(d)). The serum TNF-*α* content also increased (*P* < 0.05, Figure 1(e)). Upon comparison with the findings in the PTX 50 *μ*g/50 g group, the myocardial enzyme levels and TNF-*α* levels of the mice in the PTX 100 *μ*g/50 g and 150 *μ*g/50 g groups were increased (*P* < 0.05). These results indicate that PTX can cause different cardiac muscle damage in mice.

### 3.2. Cardiomyocyte Apoptosis after PTX Intervention

Compared with the findings in the control group (Figure 2(a)), the PTX group's apoptosis was increased (Figures 2(b)–2(d), green fluorescent dots). Compared with the findings in the PTX 50 *μ*g/50 g group (Figure 2(b)), there were apparent reductions in apoptosis after interventions with PTX 100 *μ*g/50 g and 150 *μ*g/50 g (*P* < 0.05, see Figures 2(c) and 2(d)).

RETRACTED

### 3.3. The Expression of JNK and TNF-*α* in Myocardial Tissue of Mice after PTX Intervention

The expression of TNF-*α*, JNK, and Bcl-2 family-related proteins in cardiomyocytes was also determined. Compared with the findings in the control group, the levels of JNK, TNF-*α*, p-JNK, and Bax in the PTX group were increased (*P* < 0.01). Compared with the findings in the PTX 50 *μ*g/50 g group, the interventions of PTX 100 *μ*g/50 g and 150 *μ*g/50 g reduced apoptosis (*P* < 0.01). PTX increased the protein levels of TNF-*α*, JNK, Bax, and p-JNK in cardiomyocytes, while decreasing the protein level of Bcl-2 (Figure 3).

### 3.4. The Effect of Inhibiting JNK and TNF-*α* on Mouse Myocardium after PTX Intervention

After 1 month of PTX treatment in mice, we inhibited the expression of TNF-*α* and JNK. We found that, compared with the findings in mice treated with PTX for 3 months, inhibition of TNF-*α* and JNK reduced the impact of paclitaxel on the apoptosis of mouse cardiomyocytes. In addition, the protein levels of p-JNK, Bax, and TNF-*α* in myocardial tissue cells were reduced, while the protein level of Bcl-2 was increased (see Figure 4).

## 4. Discussion

Chemotherapy is an indispensable part of antitumor therapy. Research has shown an apparent increase in the incidence of abnormal cardiac function in patients treated with chemotherapeutic drugs [22]. Therefore, there is an urgent need to clarify how to use chemotherapeutic drugs to reduce the damage to the heart and other organs. Against this background, this study examined the effect of PTX on the apoptosis of mouse cardiomyocytes, intending to identify a way of alleviating this apoptosis.

In this study, we first constructed a PTX mouse model to observe the degree of damage to the mouse myocardium caused by PTX. By determining the levels of myocardial enzymes in mice, we found that the average levels of myocardial CK, AST, CK-MB, and LDH in the mice treated with PTX were increased. At the same time, the intermediate level of serum TNF-*α* also clearly rose. This suggested that PTX can damage mouse cardiomyocytes and induce apoptosis. Further detection of TNF-*α*, JNK, and Bcl-2 family-related proteins in cardiomyocytes showed that PTX increased the protein levels of JNK, p-JNK, TNF-*α*, and Bax in cardiomyocytes and decreased the protein level of Bcl-2. This further confirmed the damaging effect of PTX on mouse cardiomyocytes and revealed that PTX could affect the protein levels of JNK and TNF-*α* in mouse cardiac tissue. Previous studies have shown that the JNK pathway is closely related to cardiomyocyte apoptosis [23]. This pathway is a branch of the MAPK pathway. When cells are stimulated, JNKK2/MKK7 or JNKK1/MKK4/SEK1 mediate the phosphorylation of Thr183 and Tyr185, which activates JNK and makes it enzymatically active [24, 25]. p-JNK can promote the expression of a variety of apoptotic proteins and regulate cell apoptosis at the mitochondrial level. Paclitaxel has been shown to promote JNK activation, ERK inactivation, and a reduction in basal p38 MAPK activity in KB-3 human epidermoid carcinoma cells [26]. As a result of a combination of several apoptotic signals, including DNA damage, oxidative stress, a deficiency of growth hormones, and radiation, mitochondrial proteins that cause apoptosis are released from the inner membrane space. JNKs have a crucial role in modifying the actions of pro- and antiapoptotic proteins found in mitochondria, in addition to the canonical nuclear signaling that results in the overexpression of proapoptotic genes and/or the downregulation of antiapoptotic genes [27, 28].

RETRACTED

Moreover, it can act on the proapoptotic protein Bax in the Bcl-2 family to induce cytochromes to enter the cytoplasm, thereby activating apoptosis. TNF-*α* activation can activate NF-*κ*B signaling, which in turn causes apoptosis [29]. JNK promotes apoptosis by blocking antiapoptotic proteins such as Bcl2 and enhancing the activities of proapoptotic proteins, particularly members of the BH3-only family of proteins. JNK is activated during microtubule-damaging agent-induced apoptosis of breast cancer cells, and active JNK is implicated in the phosphorylation of Bcl2 at Ser70 [30]. The upstream events that lead to JNK activation in response to low-dose paclitaxel treatment have yet to be studied. It has been observed that reactive oxygen species (ROS) formation is an early and critical phase in paclitaxel-induced lung cancer cell death [31].

Therefore, we speculate that inhibiting the expression of JNK or TNF-*α* can reduce the damage of PTX to mouse cardiomyocytes. In this study, after 1 month of PTX treatment in mice, we inhibited the expression of TNF-*α* and JNK proteins. We found that inhibiting TNF-*α* and JNK can decrease the effect of PTX on the apoptosis of mouse cardiomyocytes. It can reduce p-JNK, Bax, and TNF-*α* protein levels and increase Bcl-2 protein levels. It is suggested that the inhibition of the TNF-*α* and JNK signaling pathway can reduce the damage to mouse cardiomyocytes caused by PTX.

## 5. Conclusion

In conclusion, the present study revealed apparent increases in myocardial LDH, CK, CK-MB, and AST levels in mice treated with PTX. The PTX increased the protein levels of TNF-*α*, Bax, JNK, and p-JNK in cardiomyocytes while decreasing the protein level of Bcl-2. After 1 month of PTX treatment in mice, we inhibited the expression of TNF-*α* and JNK proteins. This reduced the effect of paclitaxel on the apoptosis of mouse cardiomyocytes; reduced the protein levels of TNF-*α*, p-JNK, and Bax in myocardial tissue; and caused a relative increase in Bcl-2 protein level. In summary, inhibiting the TNF-*α* and JNK signaling pathways can reduce the damage to the mouse myocardium caused by PTX. This experiment partly reveals how the damage to cardiomyocytes caused by PTX is diminished. Further, it provides ideas for preventing cardiotoxicity caused by antitumor drugs.

RETRACTED

## Figures and Tables

**Figure 1:** Changes of myocardial enzyme indexes and serum TNF-*α* in mice after paclitaxel (PTX) intervention. (a) Creatine phosphokinase (CK). (b) Muscle kinase isoenzyme (CK-MB). (c) Aspartate aminotransferase (AST). (d) Lactate dehydrogenase (LDH) level. (e) Tumor necrosis factor-alpha (TNF-*α*). ^∗∗∗^*P* < 0.0001.

**Figure 2:** Cardiomyocyte apoptosis. (a) Control group. (b) Paclitaxel (PTX) 50 *μ*g/50 g group. (c) PTX 100 *μ*g/50 g group. (d) PTX 150 *μ*g/50 g group.

**Figure 3:** The expression of c-Jun N-terminal kinase (JNK) and tumor necrosis factor (TNF-*α*) in myocardial tissue of mice after paclitaxel (PTX) intervention. (a) The expression of JNK and TNF-*α* protein in myocardial tissue. (b) The expression of JNK and TNF-*α* mRNA in myocardial tissue. ^∗^*P* < 0.05.

**Figure 4:** The effect of inhibiting c-Jun N-terminal kinase (JNK) and tumor necrosis factor (TNF-*α*) on cardiomyocyte apoptosis in mice after Paclitaxel (PTX) intervention. (a) Bax and Bcl-2 protein expression related to myocardial apoptosis. (b) The expression of Bax and Bcl-2 mRNA related to myocardial apoptosis.

## Data Availability

Data will be provided on request to authors.
